# *Butea superba* Roxb. Extract Ameliorates Scopolamine-Induced Cognitive and Memory Impairment in Aged Male Rats

**DOI:** 10.1155/2021/2703138

**Published:** 2021-10-11

**Authors:** Kittipot Sirichaiwetchakoon, Sarawut Suksuphew, Rungrudee Srisawat, Griangsak Eumkeb

**Affiliations:** ^1^School of Preclinical Sciences, Institute of Science, Suranaree University of Technology, 111 University Avenue, Suranaree Subdistrict, Muang District, Nakhon Ratchasima 30000, Thailand; ^2^Institute of Medicine, Suranaree University of Technology, 111 University Avenue, Suranaree Subdistrict, Muang District, Nakhon Ratchasima 30000, Thailand

## Abstract

*Butea superba* Roxb. (*B. superba*) is a herb that has been used for rejuvenation, to improve sexual performance, or to prevent erectile dysfunction function. Alzheimer's disease (AD) is a chronic neurodegenerative disorder that is the main cause of progressive dementia. This study aimed to investigate the amelioration for cognitive and memory dysfunction of *B. superba* ethanolic extract (BSE), a possible mechanism of action, and its toxicity. The results from the Y-maze test, novel object recognition test, and passive avoidance test exhibited that the administration of BSE at 50 mg/kg (BSL) and 200 mg/kg (BSH) could ameliorate scopolamine-induced cognitive impairment in all behavior testing. Moreover, BSE could prevent the cognitive deficit in a dose-dependent manner in a passive avoidance test. Furthermore, BSE inhibited acetylcholinesterase's (AChE) *ex vivo* activity in the cerebral cortex and hippocampus. Also, the *in vitro* and *ex vivo* antioxidative effects of BSE revealed that BSE had free radical scavenging activities in both DPPH and FRAP assay. Furthermore, male rats treated with BSE at 200 mg/kg/day for two weeks could significantly increase serum testosterone compared with control (*P* < 0.05). The GC-MS analysis and previous studies revealed that BSE contained propanoic acid, 3,3′-thiobis-, didodecyl ester, oleic acid, gamma-sitosterol, and stigmasterol which may play an important role in cognitive and memory impairment prevention. The toxicity test of BSE in rats at 50 and 200 mg/kg/day for two weeks showed that relative organ weight, serum creatinine, ALT, ALP, and CBC levels of both treated groups were not significantly different compared to the CON (*P* > 0.05). These results suggest that BSE may not be toxic to the vital organ and blood. In conclusion, BSE has the potential to be developed as a health supplement product or medicine for AD prevention and treatment.

## 1. Introduction

Alzheimer's disease (AD) is the most common chronic neurodegenerative disorder and the main cause of progressive dementia in the elderly population [1]. AD is characterized by severe memory loss, unusual behavior, personality changes, and a decline in memory function [2]. The causes of AD are still mostly unknown. However, AD is believed to occur when the neurotransmitters are deficient, resulting in progressive brain function loss. The hallmarks of AD are the deficiency of acetylcholine (ACh) and the degeneration of cholinergic neurons in the cerebral cortex and hippocampus [3–5]. Furthermore, the increase of oxidative stress in the brain may have a role in the pathogenesis of neuron degeneration and death in AD [6–8]. Also, the depletion of the sex steroid hormone testosterone was reported to increase the risk of developing AD [9, 10]. The testosterone levels have been associated with an increase in brain amyloid deposition, a main pathological feature of AD [11].

The medications that have been approved for AD by the Food and Drug Administration are AChE inhibitors (donepezil, galantamine, and rivastigmine) and N-methyl d-aspartate receptor blockers (memantine) [12]. However, these medications' efficacy is still limited, and they also provide adverse effects, such as nausea, vomiting, diarrhea, headache, dizziness, fatigue, muscle spasms, and insomnia [13]. So, the use of herbal supplements or alternative medicines instead of synthetic drugs has become increasingly popular during the last decade [14] because it may have minor adverse effects and traditional medicinal plants are often cheaper and easily consumable [15]. Many research pieces have investigated the effects of plants on inhibition of AChE, anti-inflammatory, and antioxidant activities because it may have potential in the treatment of AD [16]. Some medicinal plants such as *Emilia coccinea* [17], *Ginkgo biloba* [18], or *Melissa officinalis* [19] have been reported to alleviate cognitive and memory disorders, which may be developed to be herbal for AD treatment.

*B.superba*, a plant in the family Leguminosae, a herb used for rejuvenation, improve sexual performance, or prevent erectile dysfunction function, in Southeast Asian nations since ancient times [20]. The potential medicinal applications of *B. superba* to treat erectile dysfunction in mature human males have been reported [21]. Furthermore, it could promote penile blood flow [22] and enhance penile erection via the inhibition of cAMP phosphodiesterase activity [23, 24]. Moreover, the antioxidative activity of BSE has been reported [25] to increase serum testosterone [21, 26] and it could ameliorate cognitive and emotional deficits in olfactory bulbectomized mice by inhibiting AChE [27]. Therefore, from the evidence of BSE activities, it may potentially ameliorate cognitive and memory disorders and develop to be a health product for AD prevention.

AD is a complex multifactorial age-related neurodegenerative disorder. The naturally aged rat model is a natural animal model that provides a tractable and popular model to examine the effect of plants on age-related cognitive decline [28]. Thus, we used an aged rat model to investigate cognitive and memory impairment.

However, no work has been done about the effects and mechanism of actions of BSE on scopolamine-induced cognitive and memory impairment in an aged rat model. Although it has been reported that *B. superba* could ameliorate cognitive and emotional deficits [27], this study aimed to investigate the amelioration for cognitive and memory dysfunction in scopolamine-induced cognitive and memory impairments in aged male rats. Moreover, the chemical constituents, the possible mechanism of action, and toxicity of BSE were also studied.

## 2. Materials and Methods

### 2.1. Plant Materials

The *B. superba* ethanolic extraction was performed following the methods of Eumkeb et al. and Sirichaiwetchakoon et al. with minor modifications [20, 29, 30]. Briefly, fresh tuberous roots of *B. superba* were collected from Chiang Rai province, Thailand. Dr. Paul J Grote authenticated the plant specimen. The identification was made compared to the voucher specimen (BCU 1046) and deposited at Forest Herbarium, National Park, Wildlife, Plant Conservation Department, Ministry of Natural Resources and Environment, Thailand. The plant was washed thoroughly; then, it was ground and dried in an oven at 60°C for 72 hours (*h*). The dried powdered tuber roots of *B. superba* (2 kg) were extracted continuously with ethanol by Soxhlet extraction for 12 h. The ethanol extract was evaporated under reduced pressure to pass on the ethanol crude extract (30.5 g). The yield of the extract was 1.525 %w/w.

### 2.2. Chemicals and Reagents

Scopolamine, donepezil, acetylthiocholine iodide (ATCI), 5,5′-dithiobis (2-nitrobenzoic acid) (DTNB), 2,2-diphenyl-1-picrylhydrazyl (DPPH), 6-hydroxy-2,5,7,8-tetramethylchroman-2-carboxylic acid (Trolox), 2,4,6-tripyridyl-s-triazine (TPTZ), and ferric chloride were obtained from Sigma-Aldrich Chemical Co. (St. Louis, MO, USA). Dimethyl sulfoxide (DMSO) was obtained from Carlo Erba Reagents S.r.l. (Chaussée du Vexin, Val de Reuil, USA). All reagents used were of analytical grade.

### 2.3. Gas Chromatography-Mass Spectrometry (GC-MS) Analysis

GC-MS analyzed the active chemical compounds in *B. superba* extraction. The GC-MS analysis was performed by using Bruker Gas Chromatography Model 450 GC equipped with Bruker 320MS. The compounds were separated using an Rtx-5MS capillary column (30 m × 0.25 mm, fused silica 0.25 *μ*m). The injector volume was two *μ*L, and the injector temperature was held at 250°C. The carrier gas was helium (1 mL minute (min)^−1^). The following temperature program was set up at 40–280°C with two increasing steps. In the first step, the column oven temperature was set at 40°C for 2 min, increased to 200°C at a rate of 8°C min^−1^, and held at 200°C for 22 min. In the final step, the column oven temperature was increased up to 280°C at a rate of 5°C min^−1^. The total running time was 68 min. The compounds were identified by comparing them with NIST Mass Spectral Library.

### 2.4. Animals and Experimental Design

The animal care was designed following the method of Sirichaiwetchakoon et al. with minor modifications [30]. Accordingly, the experimental protocol of the effects, mechanism of actions, and toxicity of BSE on scopolamine-induced cognitive and memory impairment had been investigated as shown in Figure 1. Ninety 18-month-old male Wistar rats were performed for these experiments. All rats were obtained from the Animal Care Building, Suranaree University of Technology, Nakhon Ratchasima, Thailand. All rats were provided with regular food and water ad libitum and housed with 12-hour light/dark cycle, humidity, and temperature-controlled room (light on 12 h/day, temperature 25 ± 0.5°C, and the moisture 40% ± 2%) at the animal care building at the Suranaree University of Technology, Nakhon Ratchasima, Thailand. The experimental protocol was approved following a guideline for the care and use of laboratory animals by the animal care and use committee (ACUC), Suranaree University of Technology. The approval of institutional authorities on the care and use of animals number was A-2/2562.

These rats were divided into two groups. The first group was 50 rats for behavioral study. The second group was 40 rats for serum testosterone analysis, brain analysis, and toxicological testing. The treated dosage and duration of the studies were selected following the preliminary examination of each test.

### 2.5. Y-Maze Test

The Y-maze test was performed to measure general activity and basic mnemonic function. The test was executed according to Joh et al. with minor modifications [31]. Y-maze is a three-arm horizontal maze consisting of black polypropylene walls (40 cm long, 25 cm wide, and 15 cm high). The arm is symmetrically disposed at 120° angles. Before the test, rats were acclimatized to the experimental room for one week. The test relies on two phases: a sample phase trial and a test phase trial. In the sample phase trial, rats were randomly divided into five groups (*n* = 10). The control group was orally given 10% DMSO one hour before being intraperitoneally injected with sterile water for injection (CON). In the treatment group, rats were orally given 10% DMSO (SCO), BSE 50 mg/kg (BSL), and BSE 200 mg/kg (BSH) or donepezil 5 mg/kg (DNP) one hour before treatment with scopolamine (0.7 mg/kg, i.p.). Rats were initially placed in one arm one hour after treatment. The number of arm entries and the sequence (i.e., ABACB, etc.) of rats in the apparatus for 10 min were recorded. The number of actual alternations was counted by the number of entries into all three arms on consecutive choices (i.e., ABC, BCA, or CAB but not BAB). The maze was wiped clean with 70% ethanol between each animal. The sample phase trial was performed 30 min after the sample phase trial. The percentage of alternations was calculated by

(1) $$\begin{array}{c} \%\text{alternation}=\left[\frac{\left(\text{number of alternations}\right)}{\left(\text{total arm entries}-2\right)}\right]\times 100. \end{array}$$

### 2.6. Novel Object Recognition Test

This test was done following Wang et al. with minor modifications [32]. This test is based on the tendency of rats to discriminate a familiar from a new object. After Y-maze testing, rats were housed in the experimental room and regularly handled for one week prior to this experiment. Before the test, rats were habituated to the test apparatus for 5 min without objects. The test relied on two sessions: the acquisition session and the test session. The test apparatus, a black Perspex box with sawdust bedding (90 × 90 × 40 cm), was used. The acquisition session involves visual exploration of two identical objects, while the test session consists of replacing one of the previously explored items with a novel object. Acquisition session, rats were randomly divided into five groups, practically the same as the Y-maze test (*n* = 10). Briefly, rats in the control group were orally given 10% DMSO one hour before being intraperitoneally injected with sterile water for injection (CON). The treatment groups were orally given 10% DMSO (SCO), BSE 50 mg/kg (BSL), and BSE 200 mg/kg (BSH) or donepezil 5 mg/kg (DNP) one hour before treatment with scopolamine (0.7 mg/kg, i.p.). The experiment was begun one hour after the treatment. Object exploration was measured by the total time of the rat sniffed or touched each of the two objects <2 cm from its nose, and then the acquisition session was terminated, and the rats were returned to the home cage. The box was wiped clean with 70% ethanol between each animal. The test session was examined 24 h following the acquisition session. One of the two objects was replaced by an identical copy (familiar object) and a novel object. Time spent exploring each of the two items was measured and analyzed. The discrimination index (DI) was calculated by the difference between new and familiar objects exploration time divided by the sum of new and familiar objects exploration time. The formula was as follows:

(2) $$\begin{array}{c} \text{discrimination index}\left(\text{DI}\right)=\frac{\left(\text{new object}-\text{familiar object}\right)\text{exploration time}}{\left(\text{new object}+\text{familiar object}\right)\text{exploration time}}. \end{array}$$

### 2.7. Passive Avoidance Test

This learning and memory test was performed according to what was previously described [33] with little modifications. The apparatus consists of two square chambers. 80 W lamp was placed in a lighted chamber (60 × 60 × 60 cm), which was connected to a dark chamber (60 × 60 × 60 cm) with an entrance hole (15 × 15 cm). One week before this test, rats were housed in the experimental room and regularly handled for habituation. The test relies on two trials, an acquisition trial, and a retention trial. In the acquisition trial, rats were randomly divided into five groups (*n* = 10), similar to the Y-maze test. Shortly, the control group was orally given 10% DMSO one hour before being intraperitoneally injected with sterile water for injection (CON). In treatment group, rats were orally given 10% DMSO (SCO), BSE 50 mg/kg (BSL), and BSE 200 mg/kg (BSH) or donepezil 5 mg/kg (DNP) one hour before treatment with scopolamine (0.7 mg/kg, i.p.). After treatment with scopolamine for one hour, rats were initially placed in a lighted chamber. If the rats entered the dark chamber, an electrical shock (0.5 mA) was delivered to stainless steel rods for two sec. The latency time to enter the door was measured. The retention trial was performed after 24 h of the acquisition trial. The latency time of rats reentered in the dark chamber was measured up to 300 sec.

### 2.8. Brain Tissue Preparation

The rat brain tissue was prepared to assay the level of AChE, DPPH scavenging activity, and Ferric Reducing Antioxidant Power (FRAP). Rats were randomly divided into four groups (*n* = 10): (1) the control group (CON) was fed with 10% DMSO, (2) the BSE low dose (BSL) was fed with BSE at 50 mg/kg/day, (3) the BSE high dose (BSH) was fed with BSE at 200 mg/kg/day, and (4) donepezil (DNP) was fed with donepezil at 5 mg/kg/day. The experimentation was performed for two weeks. The animals were decapitated for one hour after the last administration. The skull was cut and opened, and the whole brain was immediately removed and cleaned with chilled normal saline on the ice. The cerebral cortex and hippocampus were dissected out from the brain. The frozen cerebral cortex and hippocampus were weighed and homogenized in 10 volumes of 0.1 M phosphate buffer (pH 7.4) containing 1% Triton-X-100. After centrifugation at 15000  × g and 4°C for 20 min, the clear supernatants were collected and kept at −80°C until required.

### 2.9. Ex Vivo Measurements of Acetylcholinesterase (AChE) Activity in the Brain

*Ex vivo* AChE activity in the cerebral cortex and hippocampus was determined with the colorimetric method as previously described by Ellman et al. [34]. Briefly, the assay mixture consisted of 50 *μ*L of brain homogenates, 25 *μ*L of 0.1 M phosphate buffer (pH 7.4), 125 *μ*L of 0.1 mM 5,5′-dithiobis (2-nitrobenzoic acid) (DTNB), and 25 *μ*L of 1 mM acetylthiocholine iodide (ATCI) which were mixed well. The absorbance of the assay mixture was measured by Benchmark Plus Microplate Spectrophotometer (Benchmark Plus, Bio-Rad, Japan). The spectrophotometric absorption at 405 nm during a 6 min incubation period at 25°C was quantitatively measured and was expressed as nmol ACh hydrolyzed (mg tissue)^−1^ min^−1^. The experiment was repeated six times.

### 2.10. DPPH Scavenging Activity of BSE In Vitro and Ex Vivo

The %DPPH scavenging activity of BSE was measured following Brand-Williams et al. [35] with minor modifications. *In vitro* testing, 0–1000 *μ*g mL^−1^ of BSE was prepared using methanol with a 0.02 mM DPPH solution. The samples were mixed and shaken suitably on a 96-well plate. The samples were kept in the darkroom at room temperature for 30 min. Methanol was used as the negative control, and stead of the extract was mixed with the same volume of DPPH solution in methanol as sample control. The absorbance at 515 nm was measured. The radical scavenging activity was calculated and expressed in the DPPH scavenging percentage as follows:

(3) $$\begin{array}{c} \%\text{DPPH scavenging}=\left(1\;-\;\frac{{\text{OD}}_{\text{sample}}-{\text{OD}}_{\text{sample blank}}}{{\text{OD}}_{\text{control}}-{\text{OD}}_{\text{sample blank}}}\right)\;\times \;100. \end{array}$$

Moreover, *ex vivo* testing was performed. 20 *μ*L of homogenized cerebral cortex and hippocampus samples were mixed with 0.02 mM DPPH reagent in methanol. The samples were kept in the darkroom at room temperature for 30 min. Methanol was used as the negative control, and 0.02 mM DPPH solution in methanol was used as a sample control. The absorbance at 515 nm was measured. The experiments were repeated six times.

### 2.11. FRAP Assay of BSE In Vitro and Ex Vivo

The procedure of *FRAP* assay was performed following Benzie [36] with slight modifications. This detection principle is based on reducing a ferric-tripyridyltriazine complex to its ferrous, colored form in the presence of antioxidants. Briefly, the working FRAP reagent contained 300 mM acetate buffer (pH 3.6), a solution of 10 mM TPTZ in 10 mM hydrochloric acid, and 20 mM ferric chloride at 10 : 1:1 (v/v/v). In *in vitro* testing, the BSE samples in various FRAP reagent concentrations (0–1000 *μ*g mL^−1^) were prepared and mixed in a 96-well plate for 6 min. *Ex vivo* testing, 20 *μ*L of homogenized cerebral cortex and hippocampus samples were mixed with 180 *μ*L of FRAP reagent in a 96-well plate for 6 min. The absorbance at 595 nm was measured using a microplate reader (Bio-Rad Laboratories, Inc., USA). FRAP values were calculated as a milligram of Trolox equivalent antioxidant capacity (TEAC) per Gram of dry extract. The experiments were repeated six times.

### 2.12. Serum Testosterone Analysis and Toxicological Testing

The effect of BSE on serum testosterone and toxicity experiments were investigated. Before treatment, blood was collected from all rats for measuring serum testosterone, creatinine, alanine transaminase (ALT), alkaline phosphatase (ALP), and complete blood count (CBC). Rats were randomly divided into four groups (*n* = 10) similar to brain tissue assay: (1) the control group (CON) was fed with 10% DMSO, (2) the BSE low dose (BSL) was fed with BSE at 50 mg/kg/day, (3) the BSE high dose (BSH) was provided with BSE at 200 mg/kg/day, and the positive control group, donepezil (DNP), was fed with donepezil at 5 mg/kg/day. The experimentation was performed for two weeks. At the end of the treatment, all rats were sacrificed under thiopental sodium anesthesia and subjected to necropsy. The blood was collected to analyze serum testosterone, creatinine, ALT, ALP, and CBC. Then, the liver, heart, kidney, lung, and spleen were collected, and weights were measured. The relative organ weight per 100 g of total body weight of each rat was calculated as follows:

(4) $$\begin{array}{c} \text{relative organ weight}\left(\frac{\text{g}}{100\text{ g}}\text{body weight}\right)=\frac{\text{weight of rat organ}\left(\text{g}\right)\times 100}{\text{rat body weight}\left(\text{g}\right)}. \end{array}$$

### 2.13. Statistical Analysis

All data were presented as the mean ± SEM. The statistically significant differences between groups of Y-maze test, discrimination index (DI), AChE activity, DPPH scavenging activity, and FRAP assay were analyzed by ANOVA with a Tukey's HSD post hoc test. Paired Student's *t*-test was used to compare the differences between pre- and posttreatment groups of the novel object recognition and a passive avoidance test, serum testosterone, and toxicological testing analysis. Then, a significant difference in the posttreatment group, in which baseline was adjusted for comparison, was compared using ANCOVA with Tukey's HSD post hoc test at *P* < 0.05 [26, 29, 30].

## 3. Results

### 3.1. GC-MS Analysis

The GC-MS analysis of the BSE is presented in Figure 2 and Table 1. The results showed that BSE contained 56 volatile compounds, and the abundant primary compounds were propanoic acid, 3,3′-thiobis-, didodecyl ester, and oleic acid with a %area at 13.27% and 10.36%, respectively.

### 3.2. Y-Maze Test

The Y-maze was used to examine the effects of BSE on cognitive deficits that were measured by spontaneous alternation behavior due to cholinergic dysfunction in scopolamine-treated mice. The percentage of spontaneous alternation of the scopolamine-treated group (SCO) (56.2 ± 8.15%) was significantly lower than the CON group (87.5 ± 7.14%; *P* < 0.05, Figure 3). Furthermore, both BSL and BSH groups (77.4 ± 7.58%, 79.57 ± 1.88%, respectively) showed significantly improved memory recovery from scopolamine-treated compared to CON group (87.5 ± 7.14%; *P* < 0.05, Figure 3). Interestingly, the effect of BSE, both 50 and 200 mg/kg, on the spontaneous alternation behavior was almost the same as that of the DNP group (86.25 ± 2.53; *P* > 0.05, Figure 3).

### 3.3. Novel Object Recognition Test

The effect of BSE on scopolamine-induced memory impairment in a novel object recognition test was evaluated. As a normal behavior, rats spend less time on the familiar object in the test session. In the acquisition session, rats in treatment groups were administered scopolamine or water for injection in the control group.  Figure 4(a) reveals that time exploring objects of object one and object two showed no biased exploratory preference in neither of all rat groups (*P* > 0.05). When the test session was performed 24 h after the acquisition session, Figure 4(b) displays that scopolamine caused memory impairment. The SCO group showed no difference in time exploring objects comparing the familiar and new objects (*P* > 0.05). In comparison, BSE abolished the partial amnesic effect of scopolamine. BSL, BSH, and DNP groups spent significantly more time on the new object than the familiar object within the group (*P* < 0.05) and also longer time compared to the SCO group. In the same way, Figure 4(c) reveals that the discrimination index data of BSL and BSH (0.35 ± 0.06, 0.17 ± 0.04, respectively) significantly discriminated new objects better than familiar objects compared to SCO groups (−0.075 ± 0.03; *P* < 0.05).

### 3.4. Passive Avoidance Test

A passive avoidance test investigated the protective effects of BSE on scopolamine-induced memory deficit in aged male rats.  Figure 5 displays that the retention trial of the CON group produced a significantly increased latent time to enter the dark chamber compared to the acquisition trial (27.50 ± 1.06 s, 165.75 ± 9.21 s, respectively; *P* < 0.001). The latent time of the BSH group (121.64 ± 5.06 s) was significantly longer than the BSL group (99.66 ± 4.69 s; *P* < 0.05) and not significantly different from the DNP group (126.36 ± 4.69 s; *P* > 0.05). Besides, both low- and high-dosages of BSE attenuated the harmful effects of scopolamine in a dose-dependent manner.

### 3.5. Ex Vivo Measurements of Acetylcholinesterase (AChE) Activity in the Brain

The action of BSE on *ex vivo* AChE activity in the rat brain was determined by the possible involvement of endogenous acetylcholine. The homogenated brain fraction of rats was assayed using the colorimetric method. Notably, after treating rats with BSE for two weeks, BSL and BSH groups revealed a significant decrease in AChE activity in both the cerebral cortex (0.022 ± 0.0001 nmol mg tissue^−1^.m^−1^, 0.020 ± 0.0031 nmol mg tissue^−1^.m^−1^, respectively) and hippocampus (0.012 ± 0.0005 nmol mg tissue^−1^.m^−1^, 0.010 ± 0.0029 nmol mg tissue^−1^.m^−1^, respectively) compared to control (cerebral cortex; 0.033 ± 0.0002 nmol mg tissue^−1^.m^−1^, hippocampus 0.020 ± 0.0001 nmol mg tissue^−1^.m^−1^, *P* < 0.05; Figure 6). Moreover, AChE activity in the cerebral cortex and hippocampus of BSL and BSH groups was not significantly different from the DNP group (cerebral cortex; 0.022 ± 0.0008 nmol mg tissue^−1^ m^−1^, hippocampus 0.012 ± 0.0007 nmol mg tissue^−1^ m^−1^, *P* > 0.05).

### 3.6. In Vitro Antioxidant Activities

The antioxidant activities of BSE were investigated using the DPPH radical scavenging and FRAP assay. The results showed that BSE at 0–1000 *μ*g mL^−1^ generated significantly increase antioxidant capacity, both DPPH radical scavenging and FRAP assay, with a dose-dependent manner (*P* < 0.05; Figures 7(a) and 7(b), respectively). The IC_50_ value of BSE in DPPH radical scavenging was 490.16 ± 16.47 *μ*g mL^−1^.

### 3.7. Ex Vivo Antioxidant Activities

The *ex vivo* antioxidant activities in the cerebral cortex and hippocampus after treatment with BSE for two weeks were investigated. After treating rats with BSE for two weeks, the homogenized brain fraction of rats was prepared and analyzed using DPPH radical scavenging and FRAP assay. Figures 8(a) and 8(b) reveal that the rats treated with BSE at 200 mg/kg/day significantly increased antioxidant level, %DPPH and TEAC/Protein, in the cerebral cortex and hippocampus compared to CON, BSL, and DNP groups (*P* < 0.05). Besides, the FRAP assay revealed that the BSL group in the hippocampus exhibited stronger antioxidation activities than CON and DNP groups (*P* < 0.05; Figure 8(b)).

### 3.8. Effect of BSE on Serum Testosterone

The effect of BSE on serum testosterone after treatment for two weeks is demonstrated in Figure 9. The serum testosterone of pre- and posttreated control and BSL-treated groups were not significantly different (*P* > 0.05). Also, the testosterone of ANCOVA adjusted after treatment in both groups (2.00 ± 0.19 ng dL^−1^ and 2.36 ± 0.19 ng dL^−1^, respectively) was not significantly different (*P* > 0.05). However, the serum testosterone of BSH and DNP posttreated groups was significantly higher than the pretreated groups (*P* < 0.05). In addition, the testosterone of ANCOVA adjusted after treatment in both groups (3.35 ± 0.18 ng dL^−1^ and 4.25 ± 0.20 ng dL^−1^, respectively) was considerably higher than the CON group (*P* < 0.05).

### 3.9. Effect of BSE on Relative Organ Weight

The relative organ weights of the liver, heart, kidney, lung, and spleen of rats after feeding with BSE at 50, 200 mg/kg/day and donepezil at 5 mg/kg/day for two weeks were examined. The relative weights of the liver, heart, kidney, lung, and spleen of BSL, BSH, and DNP-treated groups were not significantly different from the CON group (Table 2, *P* > 0.05). These results provide evidence that BSL, BSH, and DNP may not affect the vital organ's weight.

### 3.10. Effect of BSE on Biochemical Parameters in Serum

The toxicity of BSE on the liver, kidney, and blood after being treated for two weeks has been investigated by measuring serum creatinine, ALT, ALP, and CBC. The BSL, BSH, and DNP serum creatinine levels were not significantly different from the CON group (Figure 10(a), *P* > 0.05). These results provide evidence that BSL, BSH, and DNP may not be toxic to the kidney. Moreover, the serum ALT and ALP of the BSL-, BSH-, and DNP-treated groups were not significantly different from the CON group (*P* > 0.05, Figures 10(b) and 10(c)). These results suggest that BSL, BSH, and DNP might not be toxic to the liver. Furthermore, the CBC testing provides essential information regarding three major blood cell types, RBC and WBC count and platelets. The RBC and WBC count and platelets are shown in Figures 11(a)–11(c), respectively. These results revealed that all BSE-treated groups were not significantly different from the CON group (*P* > 0.05).

## 4. Discussion

AD is a progressive form of dementia that interferes with memory, thinking, and behavior. The leading causes of AD are believed to occur by a deficiency of acetylcholine (ACh) [3–5], the increase of oxidative stress in the brain [6–8], and the depletion of testosterone [9, 10]. Nowadays, there is no cure for AD, but the standard medication for AD treatment is donepezil. Donepezil, an AChE inhibitor, can help slow the disease's progression; however, it still lacks AD treatment efficacy.

This work's objectives were to investigate whether BSE could prevent cognitive and memory function impairments by scopolamine-induced in the aged male rats. The scopolamine model has been widely used for memory and cognitive impairment investigation. The amnesic effect of scopolamine occurs by a blockade of postsynaptic muscarinic M1 transmission, which leads to disrupting the function of the hippocampus in the working memory. The Y-maze test, novel objective recognition test, and passive avoidance test were performed for this study. Moreover, these were investigated to evaluate cholinergic system status, which correlates with functional loss in AD [37, 38].

These studies showed that BSE could ameliorate scopolamine-induced memory and cognitive impairment of all behavior testing in aged male rats. Scopolamine significantly impaired short-term spatial memory performance in the Y-maze-test. However, the efficacy of BSE on cognitive and memory amelioration was practically the same as donepezil, a standard medication. Furthermore, the novel objective recognition test result revealed that BSE could recover scopolamine-induced long-term memory impairment in a dose-dependent manner. Moreover, the passive avoidance test is one of the most frequently employed methods for evaluating memory and cognition-enhancing effects. This test revealed that BSE significantly increased memory and cognitive performance in a dose-dependent manner compared to control (*P* < 0.05). These findings are in substantial agreement with Mizuki et al. that *B. superba* alcoholic extract ameliorates cognitive deficits and depression-related behavior in olfactory bulbectomized (OBX) mice [27].

The possible mechanisms of actions on memory and cognitive impairment amelioration were investigated. One of the standard mechanisms for slowing down the progression of Alzheimer's is to inhibit the AChE enzyme. AChE enzyme can break down the neurotransmitter acetylcholine and maintain the brain's acetylcholine level, which is important for treating AD patients [39]. BSE exhibited the *ex vivo* AChE inhibition effects in the cerebral cortex and hippocampus in the aged male rats after feeding with BSE for two weeks. These results are consistent with the previous report that BSE shows 50–65% inhibitory activity on AChE [24]. The scopolamine-induced memory and cognitive amelioration of BSE suggest that it may inhibit AChE in the brain. Moreover, oxidative stress has been proposed as one factor in the pathogenesis of neuron degeneration in AD [6–8]. The studies expressed the antioxidative effects of BSE in these parts of the rat's brain. These results are consistent with Nuengchamnong et al. that an extract of *B. superba* has an antioxidative effect on the HPLC-DPPH method equipped with the MS/MS technique [25]. Besides, the depletion of testosterone is one of the leading causes of AD progression and increases AD risk, especially in older men [40]. Testosterone replacement therapy can defer the onset, slow the progression, or improve the symptoms of AD [41]. The protective effect of testosterone in AD is mediated via androgen receptors to scavenge free radicals and enhance synaptic plasticity [42]. The results of BSE-treated groups on testosterone exhibited a significant increase in the testosterone level of both BSL and BSH treated groups in a dose-dependent manner compared to the control (*P* < 0.05). These results correspond with earlier findings of Eumkeb et al. that BSE can significantly increase testosterone levels in male mice compared to the control [20, 26]. The increase of testosterone might decrease the activity of the cholinergic system and work in concert with the antagonism produced by scopolamine [43].

These findings lead us to believe that BSE may ameliorate memory and cognitive impairment by inhibition of AChE, free radical scavenging, and may slow the AD progression by preventing testosterone depletion. So, BSE may have the potential to prevent and alleviate the progression of AD.

In addition, the BSE has been identified as the main chemical constituent using the GC-MS technique. The results demonstrated that BSE contained propanoic acid, 3,3′-thiobis-, didodecyl ester, oleic acid, stigmasterol, and gamma-sitosterol. Moreover, our previous studies found that *B. superba* crude extract was isolated by column chromatography and PTLC and identified by UV-Vis, IR, Mass spectra, and NMR, containing genistein, biochanin A, and daidzein [20, 26]. Previous reports found that oleic acid supplementation and cholesterol intake restriction in an AD mouse model reduced AD-type neuropathology [44]. Besides, stigmasterol and gamma-sitosterol also showed potential in the therapy of AD [45]. Stigmasterol could induce cognitive ameliorative effects by enhancing the cholinergic neurotransmission system via the activation of estrogen or NMDA receptors [46]. Several studies have reported that genistein, one of the selective estrogen receptor modulators (SERMs), could improve brain function and memory neuroprotective effects by ameliorating amyloid beta-induced impairment [47–50]. Besides, biochanin A was reported to ameliorate behavioral and neurochemical derangements and protect memory impairment in cognitive-deficit-induced mice [51, 52]. Moreover, it exhibited neuroprotective effects by preventing beta-amyloid-induced neurotoxicity in PC12 cells via the mitochondrial-dependent apoptosis pathway [53]. Apart from this, daidzein, a polyphenolic compound in the isoflavone group was studied. It displayed potential treatment for various neurodegenerative disorders like AD by Alzheimer beta-amyloid fibril aggregation inhibition [54, 55]. These results suggest that oleic acid, stigmasterol, gamma-sitosterol, genistein, biochanin A, and daidzein in BSE may prevent memory and cognitive impairment.

Also, many compounds in BSE, stigmasterol, gamma-sitosterol, genistein, biochanin A, and daidzein, have been reported help in AChE inhibition [45, 46, 51, 56–58]. Moreover, the *in vitro* and *ex vivo* antioxidative effects of BSE may act by stigmasterol, a phytosterol, which was reported to have significant antioxidant activity, such as DPPH-, superoxide-, and hydroxyl-radical scavenging [59–61]. Besides, several researchers have reported that the isoflavones like genistein, biochanin A, and daidzein that can be found in BSE show strong antioxidant properties [62–68]. Furthermore, the depletion of testosterone is one of the leading causes of AD. Genistein, biochanin A, and daidzein have been reported to be able to significantly increase testosterone in mice [20, 69]. These findings provide evidence that oleic acid, stigmasterol, gamma-sitosterol, genistein, biochanin A, and daidzein are the main chemical constituents in BSE which may play a role in the amelioration of memory and cognitive impairment.

Besides, the toxicity test results of BSE on the relative weights of liver, heart, kidney, lung, spleen, and ALP, ALT, creatinine, RBC, WBC, and platelets revealed that these parameters of BSE-treated groups were not significantly different from the CON and DNP groups (*P* > 0.05). These results are in substantial agreement with those of Manosroi et al. where rats treated with BSE at 250 mg/kg for eight weeks appeared to be safe [70]. Apart from this, this result is consistent with earlier findings where male mice treated with 1,250 mg/kg BW/day for two weeks reveal normal histology of the heart, liver, spleen, kidney, and stomach compared to the control group [20]. However, the toxicity and safety of BSE in humans are still to be required for further investigation.

## 5. Conclusions

The present work results provide evidence that BSE can ameliorate memory and cognitive impairment on the scopolamine-induced aged rat model. Moreover, the results also showed the blood and vital organs safety after treatment with BSE. Therefore, BSE has the potential to be developed as a health supplement product for AD prevention and treatment. However, pharmacokinetics, pharmacodynamic, efficacious, and safety dose in humans are required for further studies.

## Figures and Tables

**Figure 1:** Schematic drawing of the experimental protocol. (a) The behavioral study and (b) serum testosterone analysis, brain analysis, and toxicological testing.

**Figure 2:** GC-MS chromatogram of compounds in *B. superba* extract.

**Figure 3:** Effect of BSE on the spontaneous alternation percentage in the Y-maze task. CON = 10% DMSO + sterile water i.p.; SCO = 10% DMSO + scopolamine 0.7 mg/kg i.p.; BSL = BSE at 50 mg/kg + scopolamine 0.7 mg/kg i.p.; BSH = BSE at 200 mg/kg + scopolamine 0.7 mg/kg i.p.; DNP = donepezil at 5 mg/kg + scopolamine 0.7 mg/kg i.p. Data are expressed as means ± SEM (*n* = 10). A significant difference within the group, which means sharing the different superscript letters, a, b, was compared using ANOVA and Tukey's HSD post hoc test at *P* < 0.05.

**Figure 4:** Effect of BSE on the time exploring objects in the novel objective recognition test. CON = 10% DMSO + sterile water i.p.; SCO = 10% DMSO + scopolamine 0.7 mg/kg i.p.; BSL = BSE at 50 mg/kg + scopolamine 0.7 mg/kg i.p.; BSH = BSE at 200 mg/kg + scopolamine 0.7 mg/kg i.p.; DNP = donepezil at 5 mg/kg + scopolamine 0.7 mg/kg i.p. (a) Acquisition session, (b) test session, and (c) discrimination index. Data are expressed as means ± SEM (*n* = 10). The significant difference between objects in each group was compared using paired Student's *t*-test at ^*∗*^*P* < 0.05, ^*∗∗*^*P* < 0.01, and ^*∗∗∗*^*P* < 0.001. A significant difference between ANCOVA adjusted objects in each group, which means sharing the different superscript letters, a, b, c, was compared using ANCOVA and Tukey's HSD post hoc test at *P* < 0.05. A significant difference between discrimination index in each group, which means sharing the different superscript letters, a, b, c, was compared using ANOVA and Tukey's HSD post hoc test at *P* < 0.05.

**Figure 5:** Effect of BSE on latent time in passive avoidance test. CON = 10% DMSO + sterile water i.p.; SCO = 10% DMSO + scopolamine 0.7 mg/kg i.p.; BSL = BSE at 50 mg/kg + scopolamine 0.7 mg/kg i.p.; BSH = BSE at 200 mg/kg + scopolamine 0.7 mg/kg i.p.; DNP = donepezil at 5 mg/kg + scopolamine 0.7 mg/kg i.p. Data are expressed as means ± SEM (*n* = 10). The significant differences between latent times within group were compared using paired Student's *t*-test at ^*∗∗∗*^*P* < 0.001. A significant difference between ANCOVA adjusted retention trials in each group, which means sharing the different superscript letters, a, b, c, d, was compared using ANCOVA and Tukey's HSD post hoc test at *P* < 0.05.

**Figure 6:** Effect of BSE on AChE activity in cerebral cortex and hippocampus. CON = control group; BSL = BSE at 50 mg/kg/day; BSH = BSE at 200 mg/kg/day; DNP = donepezil at 5 mg/kg/day. Data are expressed as means ± SEM (*n* = 10). The significant difference within the group was shown as different superscript letters (A, B; a, b; capital letters = cerebral cortex, lowercase letters = *hippocampus*) and was compared using ANOVA and Tukey's HSD post hoc test at *P* < 0.05.

**Figure 7:** Effect of BSE on antioxidant activities at concentrations ranging from 0 to 1000 µg mL^−1^. (a) DPPH scavenging activity assay and (b) FRAP assay. Data are expressed as means ± SEM (*n* = 6). The significant difference within the group, which means sharing the different superscript letters, a, b, c, d, and e, was compared using ANOVA and Tukey's HSD post hoc test at *P* < 0.05.

**Figure 8:** Effect of BSE on antioxidant activities in cerebral cortex and hippocampus. CON = control group; BSL = BSE at 50 mg/kg/day; BSH = BSE at 200 mg/kg/day; DNP = donepezil at 5 mg/kg/day. (a) DPPH scavenging activity assay, (b) FRAP assay. Data are expressed as means ± SEM (*n* = 6). The significant difference within the group, which means sharing the different superscript letters (A, B, C, a b, c; capital letters = cerebral cortex, lowercase letters = hippocampus), was compared using ANOVA and Tukey's HSD post hoc test at *P* < 0.05.

**Figure 9:** Effect of BSE on serum testosterone. CON = control group; BSL = BSE at 50 mg/kg/day; BSH = BSE at 200 mg/kg/day; DNP = donepezil at 5 mg/kg/day. Data are expressed as means ± SEM (*n* = 10). The significant difference between pre- and posttreatment was compared using Paired Student's *t*-test at ^*∗*^*P* < 0.05. A significant difference between ANCOVA adjusted after treatment in each group, which means sharing the different superscript letters, a, b, c, was compared using ANCOVA and Tukey's HSD post hoc test at *P* < 0.05.

**Figure 10:** Effect of BSE on biochemical parameters in serum. CON = control group; BSL = BSE at 50 mg/kg/day; BSH = BSE at 200 mg/kg/day; DNP = donepezil at 5 mg/kg/day. (a) Serum creatinine, (b) serum ALT, and (c) serum ALP. Data are expressed as means ± SEM (*n* = 10). Means with the same superscript letters, a, are not significantly different from each other (Tukey's HSD test, *P* > 0.05).

**Figure 11:** Effect of BSE on complete blood count. CON = control group; BSL = BSE at 50 mg/kg/day; BSH = BSE at 200 mg/kg/day; DNP = Donepezil at 5 mg/kg/day. (a) Red blood cell count, (b) white blood cell count, and (c) platelet count. Data are expressed as means ± SEM (*n* = 10). Means with the same superscript letters, a, are not significantly different from each other (Tukey's HSD test, *P* > 0.05).

**Table 1:** Compounds in BSE analyzed by gas chromatography-mass spectrometry (GC-MS) analysis.

Compounds	RT (min)	Area (%)
Acetic acid	3.566	2.754928
2-Propanone, 1,1-diethoxy-	5.289	1.694083
Furfural	5.7	0.967722
6-Oxa-bicyclo[3.1.0]hexan-3-one	7.32	0.567482
2,4-Dihydroxy-2,5-dimethyl-3(2H)-furan-3-one	8.237	0.203503
Benzyl chloride	8.909	0.175566
Gamma-ethoxybutyrolactone	9.899	0.184384
4H-pyran-4-one, 2,3-dihydro-3,5-dihydroxy-6-methyl-	11.615	3.771682
5-Hydroxymethylfurfural	13.468	9.711424
Phenol, 2,6-dimethoxy-	15.186	1.009532
Vanillin	16.055	0.252307
1-Dodecanol	17.059	2.20379
4-Methyl-2-oxotetrahydro-2h-pyran-4-yl acetate	17.412	3.933982
Dodecanoic acid	18.494	0.268537
Tetradecane	18.864	0.470557
Megastigmatrienone	19.467	0.153254
Lauryl acrylate	20.232	2.609731
4-((1E)-3-hydroxy-1-propenyl)-2-methoxyphenol	21.141	1.208702
Tetradecanoic acid	21.285	0.740805
Pentadecane	21.618	0.3991
Pentadecanoic acid	22.577	0.257172
Mome inositol	22.985	6.982343
1,2-Ethanediamine, N,N,N′,N′-tetraethyl-	23.317	2.788756
n-Hexadecanoic acid	24.156	8.198647
Hexadecanoic acid, ethyl ester	24.297	1.049062
Propanoic acid, 3-mercapto-, dodecyl ester	24.62	0.587247
Heptadecanoic acid	25.389	0.473218
Oleic acid	26.656	10.36139
Octadecanoic acid	26.969	1.701685
Octadecanoic acid, ethyl ester	27.203	0.318443
9-Octadecenamide	29.811	0.243337
Benzylamphetamine	31.171	0.184574
2-Dodecanone	31.885	0.228627
Glycerol beta-palmitate	31.954	0.497544
Allyl nonanoate	32.55	0.838489
Docosanoic acid, ethyl ester	33.079	0.123911
Medicarpin	33.177	0.428747
S-Indacene-1,7-dione, 2,3,5,6-tetrahydro-	33.637	0.357821
3,3,4,5,5,8-Hexamethyl-		
7-(3,4-Methylenedioxy)-tetrahydrobenzofuranone	34.212	0.198524
Anhydrovariabilin	34.399	0.30628
9-Octadecen-1-OL, (Z)-	34.513	0.52263
2-Pentadecanone	34.774	0.381615
Ethyl nonadecanoate	35.873	0.195027
Biochanin B	37.214	2.046051
Henquanin	37.423	0.392638
Coumaran-7-ol-3-one, 2-[4-methoxybenzyliene]-6-methoxy-	37.825	0.895884
4-Methylcholesta-8,24-dien-3-ol	39.03	0.150366
Cholesta-4,6-dien-3-ol, (3beta)-	39.94	0.285869
Campesterol	42.856	0.646161
Stigmasterol	43.61	1.64163
Gamma-sitosterol	45.101	3.329251
Lupenone	46.51	1.928221
Lupeol	47.237	4.036608
Tremulone	47.511	0.269601
Stigmast-4-en-3-one	48.782	0.606251
Propanoic acid, 3,3′-thiobis-, didodecyl ester	55.754	13.26531

**Table 2:** Effect of BSE on relative organ weight.

Groups	Relative weight (g/100 g body weight)				
	Liver	Heart	Kidney	Lung	Spleen
CON	2.49 ± 0.04^a^	0.22 ± 0.01^a^	0.48 ± 0.01^a^	0.44 ± 0.05^a^	0.15 ± 0.01^a^
BSL	2.31 ± 0.11^a^	0.23 ± 0.01^a^	0.49 ± 0.02^a^	0.46 ± 0.01^a^	0.16 ± 0.01^a^
BSH	2.49 ± 0.13^a^	0.23 ± 0.01^a^	0.51 ± 0.01^a^	0.39 ± 0.02^a^	0.14 ± 0.01^a^
DNP	2.56 ± 0.10^a^	0.22 ± 0.01^a^	0.51 ± 0.01^a^	0.43 ± 0.02^a^	0.16 ± 0.01^a^

CON = control group; BSL = BSE at 50 mg/kg/day; BSH = BSE at 200 mg/kg/day; DNP = donepezil at 5 mg/kg/day. Data are expressed as means ± SEM (*n* = 10). Means with the same superscript, a, in the same column are not significantly different from each other (Tukey's HSD test, *P* > 0.05).

## Data Availability

The datasets used and analyzed during the current study are available from the corresponding author upon reasonable request.
